The article "Evaluation of Antischistosomal Activities of Crude Aqueous Extracts of Artemisia annua, Nigella sativa, and Allium sativum against Schistosoma mansoni in Hamsters" was published in 2022. Journal: Biomed Res Int.

# Evaluation of Antischistosomal Activities of Crude Aqueous Extracts of *Artemisia annua*, *Nigella sativa*, and *Allium sativum* against *Schistosoma mansoni* in Hamsters

**DOI:** 10.1155/2022/5172287

**Published:** 2022-03-12

**Authors:** Yousef Abdal Jalil Fadladdin

**Affiliations:** Department of Biological Sciences, Faculty of Sciences, King Abdulaziz University, Jeddah, Saudi Arabia

## Abstract

Schistosomiasis is a neglected disease, as the World Health Organization classified it in the second category after malaria. World Health Organization approved praziquantel (PZQ) as the only chemotherapy to treat schistosomiasis. Over the years, some problems have arisen with PZQ, as it showed poor efficacy in the early stages of infection as well as the emergence of some resistance to it. In searching for new alternative drugs to treat schistosomiasis, the researchers intensified their efforts to find a new drug. The present study focuses on evaluating the effect of three plant extracts *Artemisia annua*, *Nigella sativa*, and *Allium sativum* at different doses of 31.25, 62.5, 125, 250, and, 500 *μ*g/ml; *in vitro* study was accomplished on the *Schistosoma mansoni* adult worms. The results declared that the concentration of 500, 250, and 125 of *Artemisia annua* was more effective on adult worms, and the same concentrations of *Nigella sativa and Allium sativum* gave less effect on the adult worms than the previous plant. *In vivo* study was accomplished on the hamster's tissue after exposing it to doses of the plants' extracts with different concentrations; it showed the presence of calcifications and damage to the worm eggs in the liver and spleen, as well as reducing the size of granulomas. After conducting many confirmatory studies *Artemisia annua* extract can be used as an effective and safe treatment for *Schistosoma* disease.

## 1. Introduction

The infectious diseases are caused by these five organisms: viruses, bacteria, fungi, protozoa, and helminths, infecting any other organism. There are many species of *Schistosoma*, including *Schistosoma mansoni*, that causes schistosomiasis, which is considered one of the main important infectious parasitic diseases in the tropical world. Schistosomiasis imposes a global economic and social burden compared to HIV, AIDS, tuberculosis, and malaria, due to infecting of more than 250 million people and 800 million others exposed to infection all over the world. Nevertheless, it is a neglected disease and is ranked as a second category in worldwide spreading after malaria [1]. The report issued by the World Health Organization [2] stated that the transmission of *Schistosoma* infection occurs in 78 countries, 52 of which require preventive treatment, but there is a shortage of treatment for *Schistosoma* due to the presence of only one drug treatment approved by the World Health Organization, which is praziquantel; this drug received to only 97.2 million of 290.8 million people that needed the treatment at the end of 2018 [2]. Moreover, the World Health Organization estimates that schistosomiasis is responsible for more than 200,000 deaths annually around the world [2].

Schistosomiasis is a parasitic disease of a bloodworm belonging to the genus *Schistosoma*. The genus *Schistosoma* includes six great pathogenic significances to some domestic, wild animals, and humans; intestinal schistosomiasis is caused by (*S. mekongi*, *S. japonicum*, *S. intercalatum*, *S. guineensis*, and *S. mansoni*) [3]; the latter is considered one of the most widespread endemic species in 55 countries including Egypt, the Arabian Peninsula, Sudan, Libya, sub-Saharan Africa, some Caribbean islands, and Venezuela [4], and the urogenital schistosomiasis is caused by (*S. haematobium*) which is the most predominant species being a chronic disease in fifty-three nations of the Middle East and in Africa (including Egypt) [2]. The Schistosoma differ in their types of snails (intermediate host), which they use them in their life cycle, the sites of infections in the human (definitive host), the number, and the egg shapes and sizes they produced..

Praziquantel was discovered and developed by Bayer in the 1970s and introduced to the market in 1988, a derivative compound called pyrazino-isoquinoline showed a strong efficacy on schistosomiasis. Praziquantel remains the only drug against schistosomiasis, despite more than 32 years having passed since its development; the mass drug administration (MDA) program used praziquantel as a treatment in epidemic areas in Latin America, Africa, and the Middle East [5, 6]. Further, The PZQ has a good impact against adult *Schistosoma* worms, but against the smaller stages of schistosomes, for example schistosomula; for preadult or juvenile adults, it is ineffective; in addition, it causes allergic and hypersensitivity responses and does not prevent reinfection [7]. Subsequently, duplication of treatment is in some cases vital to murder those schistosomes that have developed. Otherwise, having a sole drug to treat an illness that the effectiveness at millions of people in several geological zones is an actual worry. Hence, a new effective and safe antischistosomal drug must be developed.

Plants have long been an important source of natural products for human health. All over the world, over the past years, the antiparasite and microbial properties of plants have been verified through numerous studies, and many plants have been used as treatment alternatives due to their antiparasitic properties. Many of the compounds in medicinal plants and edible herbs have inhibited or delayed the growth of parasites, viruses, yeast/mold, and bacteria [8].

The aim of the study was to evaluate the efficacy of aqueous extract of *Artemisia annua*, *Nigella sativa*, and *Allium sativum* against *Schistosoma mansoni* (Egyptian strain) in *in vitro* as well as in golden hamsters.

## 2. Materials and Methods

### 2.1. Plant Materials

The leaves *Artemisia annua*, *Nigella sativa*, and *Allium sativum* were obtained and identified by specialists of plant taxonomy; the collected leaves of the plant were cleaned, washed well, and in the shade was dried, to prevent the loss of active ingredients, exposure to sunlight was avoided.

### 2.2. Preparation of Aqueous Extract

According to Ekpo and Etim [9] an aqueous extract was prepared from *Artemisia annua* (leaves), *Nigella sativa* (seed), and *Allium sativum* (bulbs). The dried plant parts were ground into a fine powder by an electric grinder. In two liters of distilled water, the fine powder of 200gm (1 : 10*w*/*v*) was dissolved by cold extraction and the extract was evaporated in vacuo. Using a rotary evaporator, the extract was concentrated in vacuo at a temperature of 40 °C. In a temperature-controlled oven, the extract was placed in ceramic plates inside the oven to remove residual water to give a residue weighing approximately 8.5 g at 4 °C.

### 2.3. Toxicological Study

The maximum nontoxic concentration (MNTC) was measured by applying serial dilutions of 10-300 *μ*l/m on Vero cells to test the toxicity of aqueous extracts; this was accomplished according to the Mosmann technique [10]. When the diluted extract preserves the normal Vero cell morphology and density it considered as the MNTC value when compared to untreated control cells with at least 95% of the OD.

### 2.4. Experimental Design

#### 2.4.1. Infection of the Hamster with *Schistosoma cercariae*

General anesthesia was given to the hamster at the beginning of the vital test (week 0) to lose consciousness and suppress muscle relaxation and reflex activity. Ketamine and Rompun were mixed in a 3 : 1 ratio. Intraperitoneally, 0.02 ml/30 g of hamster weight was injected. The animals were arranged on a wooden shelf and hung from the stomach area of the hamster. Cotton wool was dipped in water to allow easy penetration of the infectious phase into the skin. A 1 cm diameter metal ring was placed on each hamster. Approximately 250 cercariae were placed using the micropipette inside the metal ring to allow the cercariae to penetrate the skin [11].

#### 2.4.2. Parasite

By perfusion of the mesenteric veins and the hepatic portal system, adult *Schistosoma mansoni* worms were obtained by sacrificing eight week old infected hamsters using saline solution according to Stirewalt and Dorsey [12] technique.

#### 2.4.3. *In Vitro* Study

The in vitro study was accomplished according to Fadladdin [3] methods, where the worm perfusion was done by washing them three times with (BioWhittaker®) RPMI 1640 culture medium (Lonza, B-4800 Verviers, Belgium); this medium was used for culturing the parasite. a supplement for the medium was used; it consisted of L-glutamine (300 IU penicillin, 160𝜇g gentamycin per ml), and 20% fetal calf serum (300 𝜇g streptomycin), and antibiotics [13]. After completing the washing, 7 couples of worms were transferred to a culture plate (TPP, St. Louis, MO) in each well of the 24-well having one (ml) of the RPMI 1640 medium and one (ml) of the examined concentration (500, 250, 125, 62.5, and 31.25 *μ*g/ml) from each aqueous plant extract. So the final volume in each well was 2 (ml). The plate was incubated at 37°C in a humid atmosphere containing 5% CO_2_ (Thermo Fisher Scientific, Marietta, OH, USA) [14]. For 48 h, the parasite was kept. PZQ with a dose of 10𝜇g/ml was used as a positive control, while the negative controls with pure medium and sterile distilled water were used. All of the previous steps were performed under a sterilized laminar flow chamber. In a repeated and triplicate 3 times, the trial was carried out. The monitoring of the treated worms mating (pairing), motility rate (activity changes of worm's motor), and mortality were accomplished by using an inverted optical microscope (Olympus CK2). The worms that did not show any motility for two minutes were considered dead. Assessing the changes in the worm's motor activity (motility) of schistosomes was qualitative, and the decreased motor activity was defined as “significant” or “slight” [15]. Throughout the 48 h of the experimental incubation period, the adult schistosomes were observed, and the results were recorded at 2, 4, 6, 12, 24, and 48 h (trial endpoint for the negative control groups).

#### 2.4.4. Electron Microscope

Scanning electron microscope were used to study the morphological changes occurred on the tegument of adult male and female worms that were exposed to plant extracts at different concentrations using the Glauert technique [16].

#### 2.4.5. *In Vivo* Study

*(1) Animals*. Total of 30 experimental animals infected with *Schistosoma mansoni* were divided to 6 groups, each group consists of 5 hamsters, each hamster weighed from 105 to 130 g, and all hamsters were placed in a cages prepared for fecal material examination as follows:

(G1) Uninfected (healthy control) golden hamster

(G2) Golden hamsters infected with adult *S. mansoni* (negative control) given distill water

(G3) Golden hamsters infected with adult *S. mansoni* (positive control) oral treatment with 200 mg/kg PZQ

(G4) Adult *S. mansoni*-infected hamsters' oral treatment with 300 mg/kg *Artemisia annua*

(G5) Hamsters infected with the adult *S. mansoni* oral treatment with 500 mg/kg *Nigella sativa*

(G6) Hamsters infected with the adult *S. mansoni* oral treatment with 500 mg/kg *Allium sativum*

*(2) Histopathological Assessment*. Hamsters were slaughtered after completing the doses to obtain the liver, spleen, and kidneys, for a period of at least two weeks these organs were stored in 10% formalin. To remove excess formalin, small parts were washed overnight under running water. Slides were prepared according to Becker et al. [17] and were examined microscopically for granulomas.

*(3) Statistical analysis*. Data was analyzed by SPSS for windows version 25.0. Groups were compared using one-way ANOVA to compare quantitative data. A *p* value < 0.05 was considered statistically significant [18].

## 3. Results

### 3.1. Cytotoxicity

At the maximum nontoxic dose (MNTD) for the cytotoxicity test of the tested plant extracts (*Artemisia annua*, *Nigella sativa*, and *Allium sativum*), Vero cells showed no morphological differences compared to the control group, with values of 250, 350, and 300 *μ*l/ml, respectively.

### 3.2. *In Vitro* Study

On *S. mansoni* adult worms, the efficacy of *in vitro* treatment of aqueous extracts of *Artemisia annua*, *Nigella sativa*, and *Allium sativum* at different concentrations was studied. Movement of adult worms was decreased significantly in most concentrations. The incubation time and the concentration of the extracts were directly related to proportion in the reduction in the locomotion of the adult worms. The locomotor activity of all adult worms was monitored two hours after exposure to concentrations of 500, 250, and 125 *μ*g/ml of both *Nigella sativa* and *Allium sativum*, which showed that the motility decreased slightly.

The effect of laboratory treatment of aqueous extracts of *Artemisia annua*, *Nigella sativa*, and *Allium sativum* on *S. mansoni* adult worms (Egyptian strain) at different concentrations was investigated. Regarding motility, after exposure of adult worms to concentrations of 500, 250, and 125 *μ*g/ml of *Artemisia annua*, the movement decreased slightly, but concentrations of 62.5 and 31.25 *μ*g/ml showed a reduced movement of worms after 8 hours without complete loss of movement. While the effectiveness of *Nigella sativa* and *Allium sativum* were less than that of *Artemisia annua*, both showed a decrease in movement after 8 hours at the highest concentration. Plant extracts showed a significant decrease in worm motility at most concentrations, and this decrease was directly related to the concentration and incubation period. In the negative control group, the worms remained without change in movement for 24 hours, and their movement decreased in a period of 48 hours but did not lose the ability to move. The worms' motility decreased after being exposed to 10 *μ*g/ml of PZQ after two hours of incubation in the positive control group, while the motility was completely lost after 4 hours.

Concerning natural mating, depending mainly on the dose used and the time of exposure, the effect of all aqueous extracts on the natural mating process was effective, and the aqueous extracts caused a mating separation between the adult worm couples. *Artemisia annua* extract separated about 89% of worms in the first two hours at concentrations of 500 and 250 *μ*g/ml, 77% of schistosomes were separated after 4 hours at a concentration of 125 and 62.5 *μ*g/ml, and at the lowest concentration of 31.25 *μ*g/ml, the worms were separated by 55% after 12 hours. However, *Nigella sativa* and *Allium sativum* showed less effect than *Artemisia annua* as they showed adult worm detachment after 6 hours (62%) at high concentration (*Nigella sativa* extract was more active in separating adult worms from *Allium sativum*, but it was slightly active). The results showed that the concentrations that were not lethal to the worms were effective inhibitors of the process of natural mating. In the negative control group, the worms separated after about 12 hours of incubation. On the other hand, complete separation between worms was observed after exposure to PQZ (10 *μ*g/ml) after the first two hours of incubation in the positive control group.

The effect of aqueous extracts of *Artemisia annua*, *Nigella sativa*, and *Allium sativum* on *S. mansoni* was directly dependent on the concentration and incubation time. The extracts with the strongest effect were of *Artemisia annua*, where the concentration of 500 *μ*g/ml killed 100% (*p* < 0.001) of the adult worms after 6 hours of incubation, while concentrations of 250 and 125 *μ*g/ml of the same extract had a mortality rate of 100% on the adult worms after 12 and 24 hours of incubation, respectively (Figure 1). Although the aqueous extracts of *Nigella sativa* and *Allium sativum* at concentrations of 500, 250, and 125 *μ*g/ml, led to 100% mortality of *S. mansoni* after 12 to 24 incubation (Figures 2 and 3). The aqueous extracts showed a clear variation in the effect on adult worms, the males were more affected than females.

While the group treated with PZQ (the positive group) killed 100% of the worms after 4 hours of incubation, on the contrary, the worms remained alive for 48 hours after incubation in the untreated group, but it was less active.

### 3.3. Scanning Electron Microscope (SEM)

After incubating the adult worms with aqueous extracts of *Artemisia annua*, *Nigella sativa*, and *Allium sativum*, significant changes appeared on the tegument of *S. mansoni*. Concentrations of 500%, 250%, 125%, 62.5%, and 31.25% of the extracts showed ultramorphological variations in adult male and female worms. The extract *Artemisia annua* showed a strong effect on the morphology of the tegument of *S. mansoni* compared to the untreated groups, whereas PQZ made a complete change in the morphology of the adult worms (Figures 4(b) and 4(c)).

### 3.4. Adult Worms of *Schistosoma*

Clear morphological changes were observed in the *S. mansoni* male, since it showed some tubercles abnormalities as well as spine harms (tegument sloughing or peeling, peeling of tubercles, devastation, and spines), on its dorsal surface particularly. Also, morphological modified tubercles surrounded by bubbles were appeared, in addition of some changes or devastations in the sucker. Warping in the oral sucker was noticed in a few worms, whereas scaling, tegument wrinkling, (peeling and contraction of the dorsal area), corrosion, and sucker demolition or modifications were noticed in the females (Figures 5 and 6).

Concerning *Nigella sativa* and *Allium sativum* extracts, the worms showed similar morphological tegumental changes but of a lower degree to *Artemisia annua* stimulate morphological changes (Figure 7).

### 3.5. Histopathological Assessment

The parasite did not show a clear effect on the kidney tissues; all tissues appeared normally. While there was a clear effect on the hepatic parenchyma due to chronic granulomatosis, as well as on the spleen tissue, the granulomas consisted of many chronic inflammatory cells in the form of epithelial cells, lymphocytes, macrophages, eosinophils, and plasma cells due to numerous schistosome eggs containing miracidium in the fibrosis area (Figure 8(d)). In the spleen, the boundary between the red and white pulp was hidden and the eggs of *Schistosoma* appeared surrounded by an inflammatory cellular response. Most of the cells were dark stained, and the sinusoidal spaces were large.

When the hamsters were treated with aqueous extracts of *Artemisia annua*, *Nigella sativa*, and *Allium sativum*, the liver parenchyma cells showed moderate infiltration by chronic inflammatory cells without the presence of fibrosis area or worms' eggs (Figures 9–11). The absence of the worm eggs and fibrosis in the liver parenchyma with a significant decrease in the infiltration of chronic inflammatory cells was demonstrated. Whereas the spleen cells appeared surrounded by infiltrating lymphoepithelioid and inflammatory cells, the spleen sections displayed more or less degeneration of worm eggs.

## 4. Discussion

In the present study, aqueous plant extracts of *Artemisia annua*, *Nigella sativa*, and *Allium sativum* gave antischistosomal activity against *S. mansoni* exposed to different concentrations of 31.25, 62.5, 125, 250, and, 500 *μ*g/ml with differences in sensitivity in the *in vitro* study with respect to mating, survival time, and motility and tegumental change in adult worms; this agrees with several previous studies examined the effectiveness of plant extracts on male and female *Schistosoma* worms, where de Almeida et al. [19] did a study the on the effect of 200 *μ*g/ml of flavonoids and sesquiterpene lactones derived from *Artemisia absinthium* and *Tanacetum parthenium*, respectively on *Schistosoma mansoni*; it showed a death rate of 100% among the adult worms. de Almeida isolated parthenolide from *Tanacetum parthenium* and suggested an explanation for the mechanism of action of parthenolide on the tegument of *S. Mansoni*; he added that the *α*-methylene-*γ*-lactone material, which is found in parthenolide, interacts with the skeletal group in the nucleophiles, especially with the sulfhydryl group present in cysteine, with an addition of the Michael type. There are also cysteine residues on the tubercles and tegument surface of *Schistosoma*, in which exposed sulfhydryl interacts with parthenolide, causing morphological changes as well as disturbance or inhibition of various groups of enzymes present on the tegument of schistosomes, a similar morphological change in somewhat were obtained from the present study by using the crude extracts of *A. annua*, *N. sativa*, and *A. sativum*.

The present study has shown that the effect of aqueous extracts of *Artemisia annua*, *Nigella sativa*, and *Allium sativum* on *S. mansoni* was directly dependent on the concentration and incubation time. The strongest extracts had the effect of *A. annua*, where the concentration of 500 *μ*g/ml killed 100% (*p* < 0.001) of the adult worms after 6 hours of incubation, while concentrations of 250 and 125 *μ*g/ml of the same extract had a mortality rate of 100% on the adult worms after 12 and 24 hours of incubation, respectively. This results agree with Ferreira et al. [20] who showed the variation in the effect according to many factors such as time, dose, and type of extract when they compared alcoholic extract and aqueous extract of *Artemisia annua* from Brazil and China on *S. mansoni*. Chinese *Artemisia annua* extract at a concentration of 2 *μ*g/ml was shown to kill all worms within an hour while the same concentration in the Brazilian extract killed all worms after 17 hours of incubation, while the aqueous extract killed all worms after 17 hours of incubation.

The present study also showed that the *Nigella sativa* and *Allium sativum* at concentrations of 500, 250, and 125 *μ*g/ml, led to 100% mortality of *S. mansoni* after 12 to 24 incubation; these results are supported by Mahmoud et al. [21] who mentioned that *Nigella sativa* oil showed high activity when infected mice with *S. mansoni* worms were dosed with it. Mohamed et al. [22] reported that crushed black *Nigella* seeds had an effective effect on all stages of *Schistosoma mansoni* (Miracidia, cercariae, and the adult worms) and on egg-laying of females. The present study results showed that the garlic, or *Allium sativum* had antischistosomal activity; this agrees with Riad et al. [23] who reported that the treatment of mice with garlic reduced egg production and led to body wall damage. Nevertheless, Sutton and Haik [24] mentioned that the effect of garlic is not only the elimination of the parasite but also that garlic strengthens its host immunity to attack the parasite, and El-Shenaway et al. [25] verified this hypothesis regarding the antioxidant properties of aqueous garlic extract in the mice infected with *Schistosoma mansoni* by biochemical results. The same author mentioned that the black seed and garlic have a strong effect on schistosomiasis; it had been mentioned that garlic and onions are used to treat infections and digestive disorders.

The present study showed a significant change in the tegument of the *S. mansoni* treated with the three-plant crude extract; the changes in the tegument topography of schistosomes parasites have been used by many researchers to evaluate the activities of antischistosomal drugs, because the outer surface of *schistosoma* is a significant target for antischistosomal drugs [22, 26–30].

The present study showed that the aqueous extracts have a clear variation in the effect on adult worms, the males were more affected than females, and this result contributes to many studies which addressed that the effect on male worms was more pronounced than in females when exposed to antischistosomal drugs [30–32]. The most common explanation was that the female body is not directly connected to the host's microenvironment because most of the female body is surrounded by the gynaecophoric canal [28]. On the contrary to the present study, de Moraes et al. [33] examined the piplartine extracts against males and females of *S. mansoni* and found that there was an effect of the extract on the worms, but there is no difference in the effect between the male and female.

Severe infection with schistosomiasis leads to a change in the structure of the liver, which enhances the loss of liver function. The disease leads to liver infections in varying degrees and immune reactions until it reaches fibrosis. The chemotherapy treatment of schistosomiasis reduces egg production and prevents schistosomes from accumulating eggs in the liver, and some treatments aim to reduce, slow down, or eliminate liver fibrosis, especially in the chronic stages of schistosomiasis.

The present study showed that the parasite has a clear effect on the hepatic parenchyma due to chronic granulomatosis, as well as on the spleen tissue. The granulomas consisted of many chronic inflammatory cells in the form of epithelial cells, lymphocytes, macrophages, eosinophils, and plasma cells due to numerous schistosomes eggs containing miracidium in the fibrosis area (Figure 8(d)). In the spleen, the boundary between the red and white pulp was hidden and the eggs of *Schistosoma* appeared surrounded by an inflammatory cellular response, this is consistent with Lenzi et al. [34] who mentioned that granulomas formed by lymphocytes, mast cells, fibroblasts, reticulocytes, epithelial cells, macrophages, giant cells, eosinophils, and neutrophils in the form of a hybrid, the muscular and dynamic structure surrounding the schistosome eggs surrounded by different organs. In general, granulomas form in the intestine, lung, spleen, and liver of hamsters infected with *S. mansoni*.

The present study demonstrated that the treated hamsters with aqueous extracts *Artemisia annua*, *Nigella sativa*, and *Allium sativum*, had a positive effect on their livers as the parenchyma cells showed moderate infiltration by chronic inflammatory cells without the presence of fibrosis of the area or eggs of worms (Figures 9–11). The absence of worm eggs and fibrosis in the liver parenchyma with a significant decrease in the infiltration of chronic inflammatory cells was demonstrated; these results are constant with Mantawy et al. [35] who stated that both *Allium sativum* and *Allium cepa* had a significant decrease in egg production from the intestine and liver. The observed results also supported by Riad et al. [23] who stated that the effect of *Allium sativum* on albino mice infected with *S. mansoni* was strong and reduced egg production and granuloma size; another strong effect was obtained by treating the hamsters with these three extracts in this study that granulomas were less in number and smaller in size after histopathological examination of the liver and spleen compared to the untreated group; the observed results agreed with Riad et al. [23] and Mantawy et al. [35]. These results can be referred to reasons include that the treating extracts containing anti-inflammatory regulate nitric oxide production in macrophages and blood platelets, which destroy the parasite. For example, garlic contains mannose-bound lectin, which helps the receptors on the surface of macrophages to catch the parasite, which leads to engulf of the parasite. Garlic contains an immunomodulatory fraction, which reduces the production of Th2, which is responsible for the formation of the granuloma, and increases the production of Th1, which is responsible for resistance to the formation of the granuloma. This explanation is supported by the results obtained by previous authors, as Riad et al. [23] stated that the effect of *Allium sativum* on albino mice infected with *S. mansoni* reduced egg production and granuloma size and also increased the level of enzymes in the liver. Also, Metwally et al. [36] mentioned that the effectiveness of garlic and allicin on mice infected with *S. mansoni* has reduced worm burden cytokines and the serum concentration of liver and granuloma size.

In conclusion, the extracts of the *Allium sativum*, *Nigella sativa*, and especially *Artemisia annua* leaves can be used as an alternative and effective antischistosomal treatment against *Schistosoma mansoni*.

## Figures and Tables

**Figure 1:** Statistical analysis of the effect of *Artemisia annua* leaf aqueous extract with different concentrations and different times on the adult worms of *S. Mansoni*: (a) Conc. 500, (b) Conc. 250, (c) Conc. 125, (d) Conc. 62.5, and (e) Conc. 31.25 *μ*g/ml.

**Figure 2:** Statistical analysis of the effect of *Nigella sativa* leaves aqueous extract with different concentrations and different times on the adult worms of *S. Mansoni*: (a) Conc. 500, (b) Conc. 250, (c) Conc. 125, (d) Conc. 62.5, and (e) Conc. 31.25 *μ*g/ml.

**Figure 3:** Statistical analysis of the effect of *Allium sativum* leaf aqueous extract with different concentrations and different times on the adult worms of *S. Mansoni*: (a) Conc. 500, (b) Conc. 250, (c) Conc. 125, (d) Conc. 62.5, and (e) Conc. 31.25 *μ*g/ml.

**Figure 4:** (a) *S. mansoni* normal tegument from the hamster tissue. (b, c) Effect PZQ on adult worms of *Schistosoma*.

**Figure 5:** Effect of different concentrations of *Artemisia annua* on the tegument of *S. mansoni* by SEM. (a) Sucker destroyed (red arrows). (b–e) Male dorsal surface revealing tegumental peeling with damage and peeling of spines and tubercles (blue arrows).

**Figure 6:** Effect of different concentrations of *Nigella sativa* on the tegument of *S. mansoni* by SEM. (a) Sucker destroyed (red arrow). (b–e) Male dorsal surface revealing tegumental peeling with damage and peeling of spines and tubercles (blue arrows).

**Figure 7:** Effect of different concentrations of *Allium sativum* on the tegument of *S. mansoni* by SEM. (a) Sucker destroyed (red arrow). (b–e) Male dorsal surface revealing tegumental peeling with damage and peeling of spines and tubercles (blue arrows).

**Figure 8:** Histological section of the healthy control (negative control) and infected (untreated control) (hematoxylin and eosin staining). (a) Normal cortical structure of kidney control (×200). (b) Normal hepatic lobular structure of liver control (×200). (c) Normal structure of spleen control (×100). (d) Ova of *Schistosoma* surrounded by lymphoepithelioid tissue reaction, aggregate of deposited in the spleen (×400). (e) Multiple egg granulomas in the liver; a worm affects inside a portal vein (×400).

**Figure 9:** Histological section of treated group with 400 mg/kg *Artemisia annua*. H&E staining. (a) Inside the hepatic portal vein showing worm, radical with moderate inflammatory changes within the hepatic lobule. (b) Focal necrosis and dense inflammatory cellular reaction in liver showing enclosed intralobular ova. (c) In the spleen showing some ova surrounded by an inflammatory cellular reaction (×200).

**Figure 10:** Histological section of treated group with 600 mg/kg *Nigella sativa*. H&E staining. (a) In the liver several lymphoepithelioid granulomas. (b) In the liver merged ova granulomas (×400). (c) In the spleen several degenerated egg and fresh deposited (×200).

**Figure 11:** Histological section of treated group with 600 mg/kg *Allium satvium*. H&E staining. (a) (×200) and (b) in the liver, mononuclear inflammatory cells contained degenerated ova with mild infiltration of the hepatic lobule (×100). (c) In spleen, lymphoepithelioid cellular inflammatory cellular infiltration contained some degenerated ova (×100).

## Data Availability

The data used to support the results of this study were deposited in a repository (Twumasi et al., 2020 doi:10.1371/journal.pntd.0008919; Alves et al., doi:10.1017/S003118202000181X; Yones et al., 2016 doi:10.1155/2016/2872708; Fadladdin Y., 2021, doi:10.1155/2021/5545331).

## References

[1] Hoffmann K. F., Brindley P. J., Berriman M. (2014). Halting harmful helminths. *Science*.

[2] WHO (2020). Schistosomiasis. https://www.who.int/news-room/fact-sheets/detail/schistosomiasis.

[3] Fadladdin Y. A. J. (2021). Antischistosomal activity of *Origanum majorana*, *Ziziphus spina-christi*, and *Salvia fruticosa* plant extracts on hamster infected with *Schistosoma haematobium*. *BioMed Research International*.

[4] Barakat R. M. R. (2012). Epidemiology of Schistosomiasis in Egypt: Travel through Time: Review. *Journal of Advanced Research*.

[5] Lustigman S., Prichard R. K., Gazzinelli A. (2012). A research agenda for helminth diseases of humans: the problem of helminthiases. *PLOS Neglected Tropical Diseases*.

[6] Lo N. C., Addiss D. G., Hotez P. J. (2017). A call to strengthen the global strategy against schistosomiasis and soil- transmitted helminthiasis: the time is now. *The Lancet Infectious Diseases*.

[7] Aires A. L., Ximenes E. C. P. A., Barbosa V. X., Góes A. J. . S., Souza V. M. O., Albuquerque M. C. P. A. (2014). *β*-Lapachone: A naphthoquinone with promising antischistosomal properties in mice. *Phytomedicine*.

[8] de Moraes J., Rodriguez-Morales A. J. (2012). Antischistosomal natural compounds: present challenges for new drug screens. *Current Topics in Tropical Medicine*.

[9] Ekpo M. A., Etim P. C. (2009). Antimicrobial activity of ethanolic and aqueous extracts of *Sida acuta* on microorganisms from skin infections. *Journal of Medicinal Plants Research*.

[10] Mosmann T. (1983). Rapid colorimetric assay for cellular growth and survival: application to proliferation and cytotoxicity assays. *Journal of Immunological Methods*.

[11] Smithers S. R., Terry R. J. (1965). The infection of laboratory hosts with cercariae of *Schistosoma mansoni* and the recovery of the adult worms. *Parasitology*.

[12] Stirewalt M. A., Dorsey C. H. (1974). *Schistosoma manonsi*: Cercarial penetration of host epidermis at the ultrastructural level. *Experimental Parasitology*.

[13] Fahmy Z. H., El-Shennawy A. M., El-Komy W., Ali E., Abdel Hamid S. S. (2009). Potential antiparasitic activity of pomegranate extracts against shistosomules and mature worms of Schistosoma mansoni: in vitro and in vivo study. *Australian Journal of Basic and Applied Sciences*.

[14] Xiao S. H., Keiser J., Chollet J. (2007). In vitro and in vivo activities of synthetic trioxolanes against major human schistosome species. *Antimicrobial Agents and Chemotherapy*.

[15] Moraes J. D., Almeida A. A., Brito M. R. (2013). Anthelmintic activity of the natural compound (+)-limonene epoxide against *Schistosoma mansoni*. *Planta Medica*.

[16] Glauert A. M., Glauert A. (1974). Fixation, dehydration and embedding of biological specimens. *Practical Methods in Electron Microscopy*.

[17] Baker M., Johnson K., Roberts I. (1989). Passive arguments raised. *Linguistic Inquiry*.

[18] Snedecor G. W., Cochran W. G. (1980). *Statistical Methods*.

[19] de Almeida L. M. S., Carvalho L. S. A. ., Gazolla M. C. (2016). Flavonoids and sesquiterpene lactones from *Artemisia absinthium* and *Tanacetum parthenium* against *Schistosoma mansoni* worms. *Evidence-Based Complementary and Alternative Medicine*.

[20] Ferreira J. F. S., Peaden P., Keiser J. (2011). *In vitro* trematocidal effects of crude alcoholic extracts of *Artemisia annua*, *A. absinthium*, *Asimina triloba*, and *Fumaria officinalis*. *Parasitology Research*.

[21] Mahmoud M. R., el-Abhar H. S., Saleh S. (2002). The effect of *Nigella sativa* oil against the liver damage induced by *Schistosoma mansoni* infection in mice. *Journal of Ethnopharmacology*.

[22] Mohamed A. M., Metwally N. M., Mahmoud S. S. (2005). *Sativa* seeds against *Schistosoma mansoni* different stages. *Experimental Treatment: Memórias do Instituto Oswaldo Cruz*.

[23] Riad N. H. A., Taha H. A., Mahmoud Y. L. (2009). Effects of garlic on albino mice experimentally infected with *Schistosoma mansoni*: a parasitological and ultrastructural study. *Tropical Biomedicine*.

[24] Sutton G. A., Haik R. (1999). Efficacy of garlic as an anthelmintic in donkeys. *Israel Journal of Veterinary Medicine*.

[25] Shenaway N. S., Soliman M. F. M., Reyad S. I. (2008). The effect of antioxidant properties of aqueous garlic extract and *Nigella sativa* as anti-schistosomiasis agents in mice. *Revista do Instituto de Medicina Tropical de São Paulo*.

[26] Yones D. A., Badary D. M., Sayed H. M. B., Bayoumi S. A. H., Khalifa A. A., el-Moghazy A. M. (2016). Comparative evaluation of anthelmintic activity of edible and ornamental pomegranate ethanolic extracts against *Schistosoma mansoni*. *BioMed Research International*.

[27] Kyere-Davies G., Agyare C., Boakye Y. D., Suzuki B. M., Caffrey C. R. (2018). Effect of phenotypic screening of extracts and fractions of *Erythrophleum ivorense* leaf and stem bark on immature and adult stages of *Schistosoma mansoni*. *Journal of Parasitology Research*.

[28] Mostafa O. M. S., Soliman M. I. (2002). Experimental use of black-seed oil against *Schistosoma mansoni* in albino mice. II. surface topography of adult worms. *Egyptian Journal of Medical Laboratory Sciences*.

[29] Jiraungkoorskul W., Sahaphong S., Sobhon P., Riengrojpitak S., Kangwanrangsan N. (2005). Effects of praziquantel and artesunate on the tegument of adult *Schistosoma mekongi* harboured in mice. *Parasitology International*.

[30] Abou El-Nour M. F., Fadladdin Y. (2021). Antischistosomal activity of *Zingiber officinale*, *Piper nigrum*, and *Coriandrum sativum* aqueous plant extracts on hamster infected with *Schistosoma mansoni*. *Journal of Parasitology Research*.

[31] Shalaby I. M., Banaja A. A., Ghandour A. M. (1991). Scanning electron microscopy of the tegumental surface of in vivo treated *Schistosoma mansoni* (Saudi Arabian geographical strain) with oxamniquine and praziquantel. *Journal of the Egyptian Society of Parasitology*.

[32] Staudt U., Schmahl G., Blaschke G., Mehlhorn H. (1992). Light and scanning electron microscopy studies on the effects of the enantiomers of praziquantel and its main metabolite on *Schistosoma mansoni in vitro*. *Parasitology Research*.

[33] de Moraes J., Nascimento C., Yamaguchi L. F., Kato M. J., Nakano E. (2012). *Schistosoma mansoni*: *In vitro* schistosomicidal activity and tegumental alterations induced by piplartine on schistosomula. *Experimental Parasitology*.

[34] Lenzi H. L., Kimmel E., Schechtman H. (1998). Histoarchitecture of schistosomal granuloma development and involution: morphogenetic and biomechanical approaches. *Memórias do Instituto Oswaldo Cruz*.

[35] Mantawy M. M., Ali H. F., Rizk M. Z. (2011). Therapeutic effects of *Allium sativum* and *Allium cepa* in *Schistosoma mansoni* experimental infection. *Revista do Instituto de Medicina Tropical de São Paulo*.

[36] Metwally D. M., al-Olayan E. M., Alanazi M., Alzahrany S. B., Semlali A. (2018). Antischistosomal and anti-inflammatory activity of garlic and allicin compared with that of praziquantel *in vivo*. *BMC Complementary Medicine and Therapies*.

